# Physicochemical Properties and Antibacterial Activity of Gellan Gum Incorporating Zinc Oxide/Carbon Nanotubes Bionanocomposite Film for Wound Healing

**DOI:** 10.1155/2022/3158404

**Published:** 2022-08-28

**Authors:** Jichao Liu, Nur Arifah Ismail, Mahani Yusoff, Mohd Hasmizam Razali

**Affiliations:** ^1^Department of Hand and Foot Micro Burn Plastic Surgery, 3201 Hospital, Hanzhong 723000, China; ^2^Faculty of Science and Marine Environment, Universiti Malaysia Terengganu, Kuala Nerus 21030, Terengganu, Malaysia; ^3^Faculty of Bioengineering and Technology, Universiti Malaysia Kelantan, Jeli 17600, Kelantan, Malaysia; ^4^Advanced Materials Research Group, Faculty of Science and Marine Environment, Universiti Malaysia Terengganu, Kuala Nerus 21030, Terengganu, Malaysia

## Abstract

Wound healing dressing based on a natural polymer of gellan gum incorporating zinc oxide nanoparticles and multiwall carbon nanotubes (GG/ZnONP + MWCNT) bionanocomposite film was fabricated via the solution casting method. The physicochemical properties of the film were characterized using X-ray diffraction (XRD), Fourier transform infrared (FTIR), and scanning electron microscopy (SEM). Moreover, the antibacterial properties of the bionanocomposite film were investigated for wound healing applications. The characterization results confirmed the reinforcement of the gellan gum (GG) matrix with zinc oxide nanoparticles (ZnONP) and multiwall carbon nanotubes (MWCNT), as an amorphous GG/ZnONP + MWCNT bionanocomposite film was obtained. SEM morphological analysis shows that the addition of ZnONP and MWCNT nanofillers changed the film microstructure into a sponge-like structure that is more suitable for fluid uptake and thus more useful for wound healing. The GG/ZnONP + MWCNT bionanocomposite film demonstrated good antibacterial activity against all strains tested. Furthermore, macroscopic analysis shows that the wound treated with GG/ZnONP + MWCNT bionanocomposite film recovered completely (100%) in 14 days, compared to pure GG film (90.76%) and negative control (77.40%). As a result, the GG/ZnONP + MWCNT bionanocomposite film could be a promising wound dressing material.

## 1. Introduction

The skin is made up of three layers: the epidermis, the dermis, and the subcutaneous tissue to protect and regulate the body against physical injury [1, 2]. During daily activities, the skin was repeatedly injured, and it typically cannot heal in a short period of time with perfect regeneration and with varying degrees of scarring. In addition, certain skin injuries, such as diabetes, chronic ulcers, and severe burn wounds, may require a longer period of time to heal [3–5], necessitating intensive care to prevent serious infection and complications. Therefore, the development of medicines and wound dressing materials to speed up the healing process has become the primary focus of numerous research groups and pharmaceutical companies around the world [6–8]. Due to their biodegradability and biocompatibility, wound dressings based on natural polymer such as cellulose, chitin, chitosan, sodium alginate, and gellan gum are favored. Gellan gum (GG) was widely used for fabrication of wound dressing attributed to its high water content and soluble biopolymer, and it has strong ability to form a film or membrane to repair various organs and tissues [9–11]. Nevertheless, it is susceptible to uncontrolled material degradation and inadequate strength [12]. Recently, various metal/metal oxides like gold, silver, platinum, iron oxide, titanium oxide, zinc oxide, and so on have been incorporated to modify the chemical structure of natural polymers. According to studies, incorporating TiO_2_ and ZnO nanoparticles into natural polymer greatly improved wound healing characteristics [13, 14]. ZnO nanoparticles also exhibit unique characteristics such as great biocompatibility, low toxicity [15], strong photocatalytic activity [16], and high antibacterial properties [17], attracting our interest for usage in wound healing. Aside from inorganic ZnO nanoparticles, organic materials based on carbon component embedded in polymer are well-known methods for improving the antimicrobial activity [18, 19]. CNTs, for example, have a powerful antibacterial effect on a wide range of bacteria and viruses because they aggregate with the cells [20, 21]. Moreover, CNT antimicrobial activity can be boosted after functionalization with -OH and–COOH functional groups or hybridization with metallic compounds because they can operate as a conductive bridge over the insulating bilayer [22, 23]. CNTs in chitosan and polyvinyl alcohol (CS/PVA) polymer also worked as a reinforcing phase, improving the shape, porosity, and structural properties of CS/PVA nanofiber composites and, as a result, the cell proliferation rate. Multiple-walled carbon nanotubes (MWCNTs), in particular, increased cell survival and proliferation with minimal harmful consequences after being integrated into chitosan biopolymers [24].

It was anticipated that the combination of inorganic and organic nanofillers inserted into biopolymer would be an efficient strategy for wound healing since it promotes cell proliferation and suppresses bacterial growth in the wound. The intention of choosing and using two materials was due to their synergistic effect. Thus, it was expected that the ZnONP + MWCNT nanocomposite possessed good physiochemical properties and strong antibacterial for wound healing. Previously, the two materials of Ag/ZnO embedded in chitosan had highly light barrier characteristics and strong antibacterial and good catalytic reduction activity [25], while doped TiO_2_/MWCNT nanocomposite films revealed higher photocatalytic efficiency than single TiO_2_ as a result of the synergistic effect of TiO_2_ and MWCNTs [26]. So far, no study was reported on two materials of ZnONP + MWCNT incorporated GG biopolymer for bionanocomposite film fabrication. Therefore, in this study, the synthesized ZnONP + MWCNT composites were integrated into GG biopolymer to fabricate (GG/ZnONP + MWCNT) bionanocomposite film for wound dressing. The GG was used as the biopolymer matrix, whereas chemically synthesized ZnONP and commercial MWCNT were used as fillers. The physiochemical properties of the GG/ZnONP + MWCNT bionanocomposite film, pure GG film, and synthesized ZnONP + MWCNT nanocomposite were investigated using various instruments. The antibacterial activity of gram-positive and gram-negative bacteria commonly found in wounds was investigated. The wound healing properties of the GG/ZnONP + MWCNT bionanocomposite film were investigated in vivo.

## 2. Experiment

### 2.1. Materials

Low-acyl gellan gum (kelcogel, lot number 5C1574A) was obtained from a Huber Company, USA. Zinc nitrate hexahydrate (Mw 297.49 g/mol, CAS number 10196-18-6, product number 37796), and multiwall carbon nanotube (CAS number 306068-56-6, product number 901019) ethanol (Mw 46.07 g/mol, CAS number 64-17-5, product number 459836), citric acid (Mw 192.12 g/mol, CAS number 77-92-9, product number 251275), nitric acid (Mw 63.01 g/mol, CAS number 7697-37-2, product number 438073), glycerol (Mw 92.09 g/mol, CAS number 56-81-5, product number G7893), and calcium chloride (Mw 110.98 g/mol, CAS number 10043-52-4, product number 499609) were obtained from Sigma-Aldrich. All materials were used as received without further purification.

### 2.2. Preparation of Zinc Oxide Nanoparticles

ZnO nanoparticles were synthesized by sol-gel method using zinc nitrate hexahydrate (Zn(NO_3_)_2_.6H_2_O) as Zn^2+^ precursor. In this method, 1 g of Zn(NO_3_)_2_.6H_2_O was mixed in 20 mL of distilled water. Then, 5 g of citric acid (C_6_H_8_O_7_.H_2_O) was dissolved in 25 mL of distilled water and added dropwise to the zinc precursor solution while stirring continuously with a magnet. The gel was produced by stirring the mixed solution on a temperature-controlled magnetic hot plate stirrer at 80°C for 2 h. The obtained gel was dried at 80°C for 24 h and then calcined in a furnace at 400°C for 2 h to produce white ZnO nanoparticle powder.

### 2.3. Preparation of Zinc Oxide Nanoparticles and Carbon Nanotubes Nanocomposite

A hydrothermal method was used to create the ZnONP/MWCNT composite. Previously, commercial MWCNT was functionalized with strong acids to enhance surface hydrophilicity [27]. Generally, 0.1 g of MWCNT was sonicated in 500 mL of concentrated HNO_3_ solution (65% w/w) at 60°C for 2 h using a sonicator with 50 kHz, 200 W, and 220 V. The MWCNT were then washed with deionized (DI) water, separated from the solution via centrifugation, and dried at 60°C under vacuum for 24 h. Afterwards, 0.1 g of functionalized MWCNT was ultrasonically dispersed in 10 mL ethanol for 20 min. A solution of 0.1 g ZnO dispersed in ethanol (10 mL) was added drop by drop to the MWCNT solution while vigorously stirring at ambient temperature. To achieve a homogeneous suspension, the stirring was continued for 2 h. The suspension was placed in a stainless-steel Teflon-lined autoclave and treated for 4 h at 150°C. The resulting ZnONP + MWCNT composite was collected, washed with distilled water, and dried at 50°C overnight.

### 2.4. Preparation of Gellan Gum Incorporating Zinc Oxide Nanoparticles and Carbon Nanotubes Bionanocomposite Film

Gellan gum solution was made by dissolving 1 g gellan gum in 100 mL deionized water and continuously stirring for 2 h at 70°C. Glycerol (50 w/w%, percentage weight relative to GG) and calcium chloride (CaCl_2_) (5 mM) were added to the solution as plasticizer and binder, respectively. Then, 1 w/w% (percentage weight relative to GG) of ZnONP + MWCNT nanocomposite powder was added and stirred for 2 h. The 1 w/w% was used because it was reported that the 1w/w% nanocomposite showed the best biological and mechanical properties [28]. The nanocomposite solution was transferred to a casting dish and dried in an oven for 24 h at 50°C to produce a spherical biofilm. Prior to testing, all films were preconditioned in a desiccator (27°C, 50% RH) for at least two days. In the absence of ZnONP + MWCNT nanocomposite, a similar procedure was used to prepare pure GG biofilm. Prior to film preparation, an optimization study was conducted to determine the optimal concentration of materials required to produce a perfect biofilm [29].

### 2.5. Water Absorption Capacity of Films

The water absorption capacity of pure GG and GG/ZnONP + MWCNT bionanocomposite film was determined using the method explained by previous researcher [30, 31]. The preweighed films (25 mm × 25 mm) were individually immersed in distilled water at room temperature. Then, the soaked films were withdrawn from the medium at predetermined time interval. The swollen weights of the samples were determined by first blotting the samples with filter paper followed by accurately weighing the sample. The weights of the swollen pieces were recorded after 1, 2, 3, and 24 hours (*h*).

The water adsorption capacity (WAC) of the sample at a given time was calculated from the following formula:

(1) $$\begin{array}{c} WAC\left(\%\right)=\left(\frac{W_{s}-W_{0}}{W_{0}}\right)\times 100, \end{array}$$

where *W*_*s*_ is the weight of the sample (moist) at a given time, and W0, the initial weight of the sample.

### 2.6. Characterization

Fourier Transform Infrared Spectroscopy (FTIR) spectra were collected using a Perkin Elmer Spectrum 100 FTIR spectrophotometer with a wavelength range of 4000 to 400 cm−1. XRD analysis was performed at room temperature using a Rigaku Miniflex (II) X-ray diffractometer from 10° to 80° of 2*θ*. The morphology of films was acquired with a JOEL JSM 6360 LA scanning electron microscopy, while the size and shape of ZnONP, MWCNT, and ZnONP + MWCNT nanocomposites were observed with a Tecnai Biotwin FEI transmission electron microscopy (TEM). The surface roughness of films was analyzed using Atomic Force Microscopy (AFM), Multimode 8 ScanAsys, Bruker. A three-dimensional (3D) image of the film surface area (5 × 5 um) was obtained, and three images were captured for each sample. AFM software calculated and analyzed statistical parameters, including average roughness (Ra: average of the absolute value of the height deviations from a mean surface).

### 2.7. Antibacterial Study

Gram-positive (*Staphylococcus aureus*) and Gram-negative (*Escherichia coli*) microbes were used for an antibacterial assay. The standard growth medium (Muller-Hinton, MH, Difco™) agar was prepared by sterilising it for 15 minutes at 120°C in an autoclave. Prior to the bacterial inoculation, *Staphylococcus aureus* and *Escherichia coli* were subcultured in MH agar and incubated aerobically at 37°C for 24 h to ensure that the bacteria were in stable, contaminant-free conditions. Bacterial concentrations were determined using a simple optical density measurement on a Spectrophotometer Biomerieux Densichek Plus at 600 nm. In this study, the bacterial suspensions were adjusted to equivalent turbidity at 0.5 McFarland standards. *Staphylococcus aureus* and *Escherichia coli* inoculants were evenly distributed in sterile Petri plates containing MH agar. All bacteria were swabbed over the surface of the agar plates with a sterile cotton swab. The biofilm sample, as well as penicillin as a control, was gently pressed onto the agar. In this study, penicillin was used as a standard antibiotic for positive control. In triplicate, the plates containing film samples and agar with bacteria were incubated at 37°C for 24 h. After 24 h of incubation at 37°C, the observations on the clear zone of each plate were recorded. It is recorded as an indicator of microbial species growth.

### 2.8. Wound Healing Study

The wound healing study was tested on Sprague Dawley rats. The rats were divided into three groups: Group A: negative control (without treatment), Group B: treatment using pure GG film, and Group C: treatment using GG/ZnONP + MWCNT bionanocomposite film. In order to perform the wound healing test, a full thickness wound that extends through subcutaneous tissue on both sides at the back of the rat was created using 8.00 mm diameter of sterile biopsy punch. Each animal received two circular excision wounds on the dorsal region. Prior to the incision, the rats were given general anaesthesia. The film was applied to each animal's wound in accordance with the animal's assigned group. The wound healing process was observed at three time intervals of three, seven, and fourteen days after wounding, with three rats in each group. The wound margin area was measured with *J* image software, and the wound healing percentage (WHP) was calculated using the following formula [32]:

(2) $$\begin{array}{c} WHP=\left[\frac{\left(\text{wound area day}0\right)-\left(\text{wound area on day}X\right)}{\text{wound area day}0}\right]\;\times \;100, \end{array}$$

where *X* *=* days 3, 7, and 14 of posttrauma.

### 2.9. Ethics Statement

All methods were accomplished consistently with the pertinent guidelines and regulations, and the experiments with animal models were in line with standard guidelines. The experimental design for animal use was approved by animal ethical committee of 3201 Hospital (Approval Number 33201-2021-0121). All efforts were made to minimize animal suffering and to keep the number of animals to a minimum to demonstrate consistent effects for the procedures and treatments.

## 3. Results and Discussion

Figure 1(a) depicts photo images of pure gellan gum (GG), and gellan gum incorporating zinc oxide nanoparticles and multiwall carbon nanotubes (GG/ZnONP + MWCNT) bionanocomposite film. The diameter and thickness of both studied film nanocomposite were almost similar, at ∼ 9 cm and ∼60–70 µm, respectively. The FTIR spectra in Figure 1(b) show that the pure GG and GG/ZnONP + MWCNT bionanocomposite films had the characteristic of broad peak ranging between 3700 and 3000 cm^−1^ (max at 3300 cm^−1^) corresponding to the O-H stretching vibration modes, which should be attributed to the presence of water molecule. The next peaks, located between 2940 cm^−1^ and 2886 cm^−1^, correspond to the C-H groups, which are also present in both films [33]. The major and strong absorption peak at 1640 cm^−1^ was assigned to the *C*=*C* skeletal stretching from the GG and MWCNT compounds [34]. The peaks at 1416 cm^−1^, 1319 cm^−1^, and 1216 cm^−1^ were characteristics of the scissoring and asymmetric bending mode of CH_2_ and CH_2_ symmetric twisting, respectively, which can be observed in pure GG and GG bionanocomposite film [35]. The peaks at 1109 cm^−1^ and 1035 cm^−1^ were attributed to symmetric and asymmetric C-O-C stretching vibration, while 916 cm^−1^ and 848 cm^−1^ were the C-O stretching motion with some contribution from CH_2_ rocking, respectively [36]. The major stretching vibrations of metal oxide bond were observed at the absorption peak below 800 cm^−1^. Thus, a strong absorption peak obtained for the GG/ZnONP + MWCNT bionanocomposite film sample at 664 cm^−1^, 560 cm^−1^, and 482 cm^−1^ resembles the stretching vibration of Zn-O bonding in the crystal structure of ZnONP [37]. There were weak absorption peaks in this range (≤800 nm^−1^) for the pure GG film due to the absence of metal oxide in this sample. Additional peaks in the FTIR spectrum of the GG/ZnONP + MWCNT bionanocomposite film at 2281 cm^−1^ and 2120 cm^−1^, 1903 cm^−1^, and 1778 cm^−1^ could be attributed to C-C and *C*=*C* stretching in MWCNT, as these peaks were absent in the pure GG film sample [38].

As shown in Figure 2(a), the synthesized ZnONP is highly crystalline, as evidenced by the presence of sharp and strong peaks at 31.26°, 34.24°, 36.06°, 47.34°, 56.44°, 62.66°, 66.42°, and 67.76°, 69.08, 72.66, and 77.02, which are assigned to (100), (002), (101), (102), and (202). There are Bragg's planes in the hexagonal wurtzite structure of ZnONP [39], while commercial CNTs exhibit broad diffraction peaks at 25.8° and 42.6° (Figure 2(b)), corresponding to (002) and (100) planes, denoted the face-centered cubic (FCC) structure of the MWCNT in Joint Committee on Powder Diffraction Standards (JCPDS) No. 01–0646 [40]. Other researchers have reported similar patterns, sometimes with the presence of extra peaks due to different chirality and layers of CNTs [41]. For the film sample, broad peaks with low intensity at ∼19° and ∼22° were observed for the pure GG sample, as shown in Figure 2(c), which are characteristics of the GG compound. Numerous previous researchers reported similar findings [13, 42]. In contrast, no single peak was obtained for the GG/ZnONP + MWCNT bionanocomposite film sample (Figure 2(d)), indicating that the sample has amorphous properties. This is explained by the carbonization of organic materials that has wrapped around the surfaces of the film sample [43, 44]. The absence of the GG peaks indicates that the GG film was wrapped in a thicker layer of amorphous carbon after the addition of MWCNT. In other words, the MWCNT was widely dispersed on the surface of the nanocomposites film, resulting in the amorphous property of the film sample. Furthermore, no peaks attributed to the MWCNT or ZnONP fillers appear in the XRD pattern, indicating that the fillers have been completely dissolved in the nanocomposites film [45, 46]. The amorphous features of the bionanocomposite film sample were expected since the presence of ZnONP and MWCNT nanofillers causes the random ordering of the GG chain matrix. They were categorized as a short-range order of repeating units with nonuniformly packed molecules, which contributed to the flexibility and elasticity of the bionanocomposite film [47].

Figure 3 shows TEM images of the synthesized ZnONP, commercial MWCNTs, and ZnONP + MWCNT nanocomposite. ZnO nanoparticles had a nearly spherical shape with a diameter of 17.31 ± 3.79 nm (Figure 3(a)), whereas MWCNT samples (Figure 3(b)) had elongated hollow nanostructures. The nanotube diameter was determined to be 9.32 ± 1.62 nm. Interestingly, the nanocomposite of ZnONP + MWCNT was successfully synthesized in this study, as both spherical shape nanoparticles and hollow elongated structures of nanotubes could be seen in the TEM image (Figure 3(c). However, the diameters of the ZnONP and MWCNT were slightly larger, at 20.57 ± 4.78 nm and 11.11 ± 1.62 nm, respectively, due to crystal growth during the hydrothermal reaction that produced the nanocomposite.

SEM was used to examine the surface morphology of the GG/ZnONP + MWCNT bionanocomposite film. The surface image of pure GG film was also studied for comparison. Due to the homogeneously blended biopolymer, a smooth and continuous surface of pure GG film was observed, as shown in Figure 4(a). However, due to the presence of nanostructure fillers, the formation of clusters on the GG/ZnONP + MWCNT bionanocomposite film was visible, indicating that ZnONPs + MWCNT were successfully loaded onto film. Even so, the nanostructures were agglomerated to reduce surface energy because ZnONP and MWCNT have high surface energy when they are nanosized within the polymer matrix [48, 49]. Different shapes of ZnONP and MWCNT fillers also promote agglomeration via an interlocking mechanism [50]. The interlocking phenomenon, which helps particles stay together in a conglomerate, is related to the shape of the particles and how they mechanically block each other's movement at the particle level. Long MWCNT particles can interlock with spherical ZnO nanoparticles and restrain their movement in this case. Thus, in Figure 4(b), an agglomeration of ZnONP + MWCNT nanocomposite can be seen, as well as the presence of the interconnected pores' structure. The porous structure of the GG/ZnONP + CNT bionanocomposite film was thought to be formed by the agglomeration of ZnONP + MWCNT nanostructures.  Figure 5 depicts cross section SEM micrographs of cold-fractured films. The essential asymmetric nature of the film, with a dense top layer, and the sublayer was observed at bottom of pure GG film (Figure 5(a)), while for the GG/ZnONP + CNT bionanocomposite film, a sponge-like pore structure was observed suggesting that pores were fully developed in the bionanocomposite film. The pores were nearly spherical and similar in size, measuring approximately 10.60 ± 2.53 µm in diameter (Figure 5(b)). In theory, the formation of interconnected pores' structure allows cell migration or tissue invasion from pore to pore [51–53].

Water absorption capability of the film is important to prevent dehydration of tissue, inhibit microorganism growth, and also protect wound maceration [31]. As stated in Table 1, the water absorption capacities of GG and GG/ZnONP + MWCNT bionanocomposite films were increased over the period of time studied. Apart from this, it also showed that GG/ZnONP + MWCNT had the higher water absorption capacity than pure GG biofilm. It is expected that, due to hydrophilic nature and water holding capacity of ZnO and MWCNT, thus, it enhances the water absorption capacity of the bionanocomposite film.

Due to their poor compatibility with the GG polymer matrix, ZnONP + MWCNT nanocomposite fillers are also unevenly distributed on the surface. Agglomeration and nonhomogeneous distribution of the ZnONP and MWCNT contributed to the higher surface roughness of the GG/ZnONP + MWCNT bionanocomposite film compared to pure GG biofilm. The roughness value (*R*_*a*_) was determined to be 9.93 ± 0.03 nm for pure GG and 19.60 ± 0.20 nm for GG/ZnONP + MWCNT bionanocomposite films, respectively. The findings suggest that incorporating ZnONP + MWCNT nanocomposite fillers into GG polymer matrix could alter the surface topography, thereby affecting roughness.  Figure 6 shows the three-dimensional (3D) AFM topography images of the film surfaces. As seen, the structures of the film surfaces are represented as dark and bright valleys and peaks, respectively. Pure GG biofilm has a flat surface with a large amount of dark area and a small amount of bright area (Figure 6(a)). In contrast, the presence of many peaks and brighter sites on the GG/ZnONPs + MWCNTs film confirms the presence of ZnONP + MWCNT nanocomposite on the film surface. Due to their increased roughness, the valley-like structure and surface ridges are clearly visible in the image of the GG/ZnONP + MWCNT bionanocomposite film (Figure 6(b)). The deep valley of the film and the height of its surface ridges contributed to the film's greater roughness [54, 55].

As shown in Figure 7, after 24 h of incubation, pure GG biofilm exhibited no antibacterial activity against any of the bacteria studied. Intriguingly, the incorporation of ZnONP + MWCNT nanocomposite into GG film yields positive results, with the GG/ZnONP + MWCNT bionanocomposite film exhibiting inhibition zones. The exhibition zones against *Staphylococcus aureus, Streptococcus, Escherichia coli*, and *Pseudomonas aeruginosa* were found to be 10 ± 0.38 mm, 12 ± 0.06 mm, 11 ± 0.06 mm, and 10 ± 0.12 mm, respectively. The antibacterial activity of pure GG biofilm, GG/ZnONP + MWCNT bionanocomposite film, and penicillin as a control sample was summarized in Table 2. The results show that GG/ZnONP + MWCNT is a promising antibacterial film because its antimicrobial activity is comparable to or better than the control sample (penicillin), ZnONP and MWCNT as separated materials.

The synergy antibacterial effect of ZnONP and MWCNT supports the good performance of the GG/ZnONP + MWCNT bionanocomposite film in exhibiting bacteria growth. The antimicrobial properties of ZnO are based on the electrostatic interaction between the nanoparticles and the microbial cell surface, which causes photodestruction via oxidative damage [58]. Furthermore, their high efficiency in inhibiting the growth of pathogen microorganisms even at very low concentrations is due to the formation of reactive oxygen species (ROS) such as HOO•, HO•, •O_2_^−^, and H_2_O_2_ via redox reactions. The inclusion of MWCNT enhances ROS generation via chemical interactions between the latter and the surface of microorganisms [59]. MWCNTs also have a large surface area, which makes them an excellent base material for photocatalytic functionalization. There is a combination with a photocatalytic agent of ZnO to form nanocomposites with antimicrobial activity under solar light irradiation [60–62]. Due to the good electrical conductivity and photothermal activity of MWCNT, the ZnONP + MWCNT nanocomposite in GG could produce photo-induced electron for photocatalytic degradation of bacteria [63, 64].

The wound healing experiment was carried out on *Sprague Dawley* rats using pure GG and GG/ZnONP + MWCNT bionanocomposite films. For comparison, a control sample in which the wound was cleaned with distilled water was also examined. Wound healing was observed on days 3, 7, and 14 following treatment, and photo images obtained are shown in Figure 8. The wounds treated with GG and GG/ZnONP + MWCNT bionanocomposite films appeared to be dried with the scab generated on the third day, whereas wounds in the control sample were found to be moist due to the lack of exudates. On the seventh day, granulation tissue formation was clearly visible on wounds treated with GG/ZnONP + MWCNT nanocomposite and pure GG films. The control sample had no granulation tissue. The open wounds for the samples treated with GG film and the control were still visible on day 14. Otherwise, the wound treated with the GG/ZnONP + MWCNT bionanocomposite film healed completely, and the damaged skin was repaired.

Figure 9 shows that a wound treated with GG/ZnONP + MWCNT bionanocomposite film healed completely (100% recovered) after 14 days. In contrast, wound contraction rates of 90.76% and 77.40% were calculated for wounds treated with pure GG film and control samples, respectively. Previously, at the seventh day, wound contraction was 82.67%, 64.71%, and 53.95% for treatments with GG/ZnONP + MWCNT nanocomposite, pure GG films, and control sample, respectively. On the third day, the smaller wound contraction was obtained with 59.82%, 44.54%, and 42.86% for each treatment. The results showed that the GG/ZnONP + MWCNT bionanocomposite film has better wound healing ability than pure GG film and control sample, as the wounds on *Sprague Dawley* rats were fully recovered with no scar. In fact, hair is regrowing to conceal the injury. The interconnected pores' structure of the GG/ZnONP + MWCNT bionanocomposite film provides a pathway for the exchange of nutrients within the temporary structure for tissue regeneration [65]. Furthermore, the interconnected pores of the GG/ZnONP + MWCNT bionanocomposite film, which has a sponge-like structure, are excellent for fluid uptake, which is advantageous in wound healing dressing applications. According to the researchers, the interconnected porous structure facilitates tissue regeneration by allowing the introduction of mesenchymal cells, osteotropic agents, or vasculature into the pores [53]. Moreover, the morphology of MWCNT in bionanocomposite film, which mimics the fibrillar/extracellular matrix protein, promotes tissue regeneration and wound healing [66]. On top of that, the antibacterial properties of the GG/ZnONP + MWCNT bionanocomposite film against bacteria such as *Staphylococcus aureus*, *Streptococcus*, *Escherichia coli*, and *Pseudomonas aeruginosa*, which are commonly found in wounds, help speed up the healing process. As a result, the wound could heal faster and without scarring. The GG/ZnONP + MWCNT work well as antibacterial and wound healing when they are combined due to their synergetic effect. It was reported that pristine ZnO exhibits good antibacterial activity that is nontoxic and biocompatible to human cells [67]. While the ZnO based wound dressing film facilitates angiogenesis, it enhances the vascular endothelial growth factor (VEGF) and hypoxia inducible factor (HIF-1*α*) [68]. Researchers reported that the modified ZnO quantum dots and hydrogel loaded with heparinized ZnO enhanced the healing rate up to more than 90% after 14 days of treatment [69, 70]. The same goes to the MWCNT film, and a good healing activity was observed after 14 to 21 days. The histological analysis further confirmed the enhanced epithelization and faster regeneration in the MWCNT nanocomposite treated group [71]. The well-formed highly vascular granulation tissue in MWCNT treated group showed a better healing activity by the composite as compared to pristine sample. The antibacterial performance of the MWCNT composite also contributes to the accelerated wound closure [72]. Both materials ZnO and MWCNT show good antibacterial properties and wound healing; thus, the synergy effect of these materials in GG biofilm enhanced the antibacterial properties and wound healing performance of the GG/ZnONP + MWCNT bionanocomposite film.

The ultrasound image of the healed wound area on the 14^th^ day after creation was obtained by using a real-time high resolution 20 MHz ultrasound DermaLab Combo, Cortes, Denmark, as shown in Figure 10. The wound treated with GG/ZnONP + MWCNT bionanocomposite film shows the formation of clear and thicker dermis, epidermis, and subcutis layers as compared to control and GG biofilm. This is probably because the amount of collagen expression in the wounds treated by the bionanocomposite film wound dressing is ideal and more than the collagen expression in the control group and pure biofilm [73].

## 4. Conclusion

A GG/ZnONP + MWCNT bionanocomposite film was successfully prepared using the solvent-casting method. The physicochemical properties of the film were studied using FTIR, XRD, SEM, and AFM. Wound healing experiments were conducted in vitro and in vivo with 3T3 mouse fibroblast cells and *Sprague Dawley* rats, respectively. The main functional groups of GG, ZnONP, and MWCNT were detected in the bionanocomposite film's FTIR spectra. The XRD pattern reveals an amorphous bionanocomposite film, indicating that the ZnONP and MWCNT nanocomposite were successfully dispersed onto the GG film. Due to their smaller size, the nanocomposite agglomerated, creating the interconnected pore structures in the GG/ZnONP + MWCNT bionanocomposite film. As nanofillers, ZnONP and MWCNT increased the roughness of the GG/ZnONP + MWCNT film, thereby promoting cell proliferation and wound healing. The wound healing rate was 100% after 14 days of treatment with GG/ZnONP + MWCNT bionanocomposite film. Furthermore, the synergy antibacterial effect of ZnONP and MWCNT supports the good performance of the GG/ZnONP + MWCNT bionanocomposite film for wound healing.

## Figures and Tables

**Figure 1:** (a) The photo images and (b) FTIR spectra of pure GG film and GG/ZnONP + MWCNT bionanocomposite film.

**Figure 2:** XRD pattern of (a) ZnONP, (b) MWCNT, (c) GG film, (d) GG/ZnONP + MWCNT bionanocomposite film.

**Figure 3:** TEM images of (a) ZnONP, (b) MWCNT, and (c) ZnONP + MWCNT nanocomposites.

**Figure 4:** SEM images of (a) GG film and (b) GG/ZnONP + MWCNT bionanocomposite film.

**Figure 5:** Cross-section SEM images of (a) GG film and (b) GG/ZnONP + MWCNT bionanocomposite film.

**Figure 6:** Three-dimensional (3D) height images of AFM of (a) pure GG film and (b) GG/ZnONP + MWCNT bionanocomposite film.

**Figure 7:** Agar well diffusion test results of control sample (penicillin), pure GG, and GG/ZnONP + MWCNT bionanocomposite films against (a) *Staphylococcus aureus*, (b) *Streptococcus*, (c) *Escherichia coli*, and (d) *Pseudomonas aeruginosa* bacteria.

**Figure 8:** Macroscopic examination of untreated wounds as control sample and treated with pure GG and GG/ZnONP + MWCNT bionanocomposite films on 3^rd^, 7^th^, and 14^th^ days.

**Figure 9:** Wound healing percentage of the untreated wound (control) and treated with pure GG and GG/ZnONP + MWCNT bionanocomposite films at 3^rd^, 7^th^, and 14^th^ days on Sprague Dawley rats. The presented data are expressed with mean ± SD, *n* = 6). Statistical analysis using one-way ANOVA followed by post hoc test shown by different letters (a, b) was statistically different (*P* ≤ 0.05).

**Figure 10:** Ultrasound images of healed wound area on Sprague Dawley rats treated with (a) control, (b) GG, (c) GG/ZnONP + WMCNT on day 14.

**Table 1:** Water absorption capacity analysis for GG and GG/ZnONP + MWCNT bionanocomposite film (mean ± SD) (*n* = 3).

Sample	Water absorption (%)			
	After 1 h	After 2 h	After 3 h	After 24 h
GG	680 ± 22	722 ± 28	884 ± 26	906 ± 24
GG/ZnONP + MWCNT	948 ± 26	1182 ± 24	1226 ± 28	1250 ± 28

**Table 2:** Inhibition zone of biofilms against Gram-positive and Gram-negative bacteria (mean ± SD) (*n* = 3).

Sample	Diameter of Inhibition (mm)			
	*Staphylococcus aureus*	*Streptococcus*	*Escherichia coli*	*Pseudomonas aeruginosa*
Penicillin	12 ± 0.06	12 ± 0.06	10 ± 0.12	9 ± 0.06
GG	0 ± 0	0 ± 0	0 ± 0	0 ± 0
GG/ZnONP + MWCNT	14 ± 0.25	14 ± 0.10	14 ± 0.05	11 ± 0.07
ZnONP [56]	14 ± 1.0	n.a	9 ± 2.0	8 ± 3.0
MWCNT [57]	0 ± 0	n.a	11.3 ± 0.3	0 ± 0

^*∗*^n.a = data not available.

## Data Availability

The data used to support the findings of this study are included in the article.
